# Multimodal Orbital Angular Momentum Data Model Based on Mechanically Reconfigurable Arrays and Neural Networks

**DOI:** 10.1155/2022/3224490

**Published:** 2022-06-23

**Authors:** Lijun Zhang, Shaojin Wang, Xinhua Zhu, Xiaohui Guo, Yuanbing Gu

**Affiliations:** School of Northwest A & F University, Yangling, Shaanxi 712100, China

## Abstract

Multimodal orbital angular momentum is a research hotspot in the field of electromagnetic wave communication. How to accurately detect and identify multimodal orbital angular momentum data is a current academic problem. Based on the theory of mechanically reconfigurable arrays and neural networks, the purity, detection method, and transmission and reception of orbital angular momentum vortex waves are modeled in this paper. Through the network identification of the dynamic model of the three-degree-of-freedom reconfigurable manipulator, the paper takes the identification result and the control input of the single neuron PID as the input of the system control torque of the manipulator and realizes the reconfigurable manipulator. In the simulation process, the local approximation effect of the nonlinear control system used is very ideal. The single neuron PID controller overcomes the shortcomings of time-consuming and unsatisfactory control accuracy caused by the constant parameter of the traditional PID controller and realizes the circular loop. On the other hand, at the point of interest of the human eye, its resolution value is the largest, and its value gradually decreases as the distance from the pit increases. The experimental results show that the three-transmitting and three-receiving orbital angular momentum vortex wave transceiver system based on the mechanically reconfigurable array and neural network theory is relatively complete, and the transmission coefficient between the same modes reaches 0.827, which is much higher than that between different modes. On this basis, the modal purity, detection method, and reception of orbital angular momentum are studied accordingly. At the same time, the damage to the microscopic particles can be greatly reduced. At the same time, the information delay is reduced to 8.25%, which effectively improves the isolation characteristics of different modal orbital angular momentum channels and promotes the communication transmission of multimodal signals.

## 1. Introduction

With the continuous development of industrial productivity, people's lives have begun to become intelligent, robots have entered the social industry and people's lives, and reconfigurable robots have also attracted people's attention. The reconfigurable robot has the double repeatability of the mechanical system and the control system, and the completed tasks are no longer single and unchanged, which reduces the use cost of the robot and greatly improves the efficiency [1–3]. The research content of this paper mainly includes kinematics analysis and dynamics research of reconfigurable robots, as well as neural network PID motion control and simulation research of reconfigurable robots. In addition, during this period, with the promotion of high-bandwidth application technology, a lot of research work focused on the polarization, amplitude, and phase multiplexing of the optical field, which also increased the data more or less transmission efficiency [4–6]. Due to the continuous breakthrough of various technologies, the channel capacity based on single-mode fiber (SMF) is getting closer and closer to the Shannon capacity limit. The computational model enhances target contours in natural scenes while suppressing irrelevant environmental elements, thereby realizing the saliency extraction of target contours. The OAM multiplexing technology of vortex beams is introduced into wireless optical communication, which can be organically integrated with MIMO technology. However, according to recent related optical communication surveys, with the development and progress of society, optical fiber communication is facing a more and more prominent key problem, that is, the existing optical communication capabilities are gradually unable to meet the increasing demand for communication capacity [7–11].

However, the helical parabolic antenna structure used in the experiment is a single fixed structure, and this single structure cannot generate multiple OAM modes at the same time. Due to the advent of the era of big data and the rapid development of wireless communication, people's demand for wireless communication is increasing day by day. The way of wireless communication technology to realize information transmission is to carry information transmission through electromagnetic waves. In order to prevent the electromagnetic waves from each other, people need to constantly expand the frequency band used. However, spectrum resources are increasingly tight, and channel capacity is becoming Shannon's limit. Therefore, the change in reuse technology is particularly important [12]. The orbital angular momentum vortex wave has a helical wavefront phase. Since the orbital angular momentum vortex wave between different modes is orthogonal to each other, and theoretically the orbital angular momentum vortex wave has infinitely many modes, the orbital angular momentum vortex wave has an infinite number of modes. The number of modes of the swirl wave is used as a modulation parameter, and the information of each channel is modulated on the orbital angular momentum vortex wave of different modes so that under the same carrier frequency, there will be infinitely many independent orbital angular momentum channels, using the orbital angular momentum vortex. Therefore, some people think that the orbital angular momentum multiplexing technology is expected to become the transmission technology adopted by the next-generation mobile communication system [13–15].

Firstly, the kinematics analysis and model establishment of the reconfigurable manipulator are carried out in this paper, and the simulation verification is carried out. At the same time, due to the nature of the orbital angular momentum vortex wave itself, the vortex waves of different modes are mutually orthogonal, so the three-way signals are independent of each other and do not interfere with each other. The general formula of forward kinematics of each module of the reconfigurable manipulator is proposed, and this formula is applicable to the four types of modules of the manipulator. Finally, according to the mechanical configuration of the robotic arm, MATLAB Robotics Toolbox is used to obtain the position and attitude and verify it. The inverse kinematics solution method of the configuration plane division method is proposed to solve the joint angle of each joint module of the reconfigurable manipulator under the condition of known working point. Second, the dynamics of the six-degree-of-freedom reconfigurable manipulator is modeled. Still citing the concept and division method of the configuration plane, the traditional dynamics are divided into the dynamic analysis between the configuration planes and the dynamic analysis in the configuration plane. The simulation results of the dynamic model obtained by the Newton–Eulerian recursion method of dividing the configuration plane are compared with the modeling results of the traditional Newton–Eulerian method. In addition, two frequency bands and two modes of OAM vortex waves are generated by using the inner and outer ring array antennas, but the far-field pattern of the high-frequency band is not very ideal, and further research is needed to reduce the outer ring as much as possible for the effect of the antenna on the inner ring antenna.

## 2. Related Work

In recent years, in industrial, life, and other production applications, the most easily accepted and widely used controller is the PID-type controller. However, due to changes in the relevant parameters of the system, or changes in disturbances and payloads during the control process, the parameters of the PID controller need to be optimized to provide a suitable and stable control law for the controlled system. The parameters in the traditional PID controller are constant, the system takes a long time to stabilize during the control process, and the robustness of the system output is not high. However, researchers have found that neural networks have excellent learning ability, which creates a new way to find faster and more robust adaptive controllers to adapt to disturbances and changes in related parameters and models during the control process and the impact caused by uncertainty [16–18].

Iakovidis et al. [19] found that, at the information sending end, the ordinary electromagnetic wave carrying information is passed through the stepped reflecting surface (assuming that the modal number of the orbital angular momentum generated by the reflecting surface is l) so that the azimuth angle is added with a rotation of 2 phase, thereby twisting ordinary electromagnetic waves propagating in phase on the plane into orbital angular momentum vortex waves of helical phase wavefronts. Ebrahimi et al. [20] believe that at the information receiving end, the received orbital angular momentum electromagnetic vortex wave passes through another stepped reflecting surface, and the modal number of orbital angular momentum generated by the reflecting surface is -1. If the angle is reversed by l, the orbital angular momentum vortex wave can be restored to the ordinary electromagnetic wave. In the first column of the signal transmitting end, modulate 4 channels of signals to 4 channels of ordinary electromagnetic waves of the same carrier frequency. Zamani Kouhpanji and Stadler [21] analyzed it and then due to the orbital angular momentum vortices of different modes, the ordinary Gaussian electromagnetic wave is converted into four vortex electromagnetic waves with different modes by phase rotation. The waves are orthogonal to each other, so on the premise of multiplexing the orbital angular momentum vortex wave mode *l*, polarization multiplexing is introduced at the same time, that is, different polarization directions are arranged for the orbital angular momentum channels of each mode, then at the same frequency, on the other hand, the use of 4 polarization multiplexed orbital angular momentum vortex wave channels can transmit 8 channels of information and can ensure that these 8 channels of information do not interfere with each other. Chang et al. [22] found that at the signal reception, we rotate the orbital angular momentum vortex wave signal of a specific mode in the opposite phase and then use the orthogonality of the orbital angular momentum vortex wave itself to convert a certain mode The orbital angular momentum vortex wave signal of *l* is restored to the ordinary signal, and the demultiplexing of the orbital angular momentum signal is realized.

This scheme is based on the equivalent medium theory. Applying this concept to 2D metasurfaces, Tang et al. [23] proposed encoding metasurfaces to simplify the design of metasurfaces. Coded metasurfaces can be used to achieve transmission and reflection beamforming, radar cross section reduction, phase gradient surfaces, invisibility cloaks, and absorbers. By loading active devices on the encoded metasurfaces, digital metasurfaces can be formed. These applications of encoding metasurfaces are based on the generalized reflection and refraction theory, which states that abrupt phases of surfaces can shape beams. In this section, we propose a 1-bit digital orbital angular momentum vortex generator to simplify the generation of vortex waves in the radio frequency domain, based on the theory of coded artificial metasurfaces for regulating electromagnetic waves. The concept of digitization is widely used in the field of electronic engineering, but its application to the field of microwave and optics has encountered resistance because the operating wavelength of microwave and optical components is usually comparable to the size of individual components [24, 25].

## 3. Mechanically Reconfigurable Arrays and Neural Network Data Sets

### 3.1. Reconfigurable Array Regular Matrix

When the effective refractive index difference between modes in a reconfigurable array is less than 10′4, they undergo mode degeneracy as they propagate and form scalar LP modes. However, after the scalar LP mode is transmitted over a long distance, due to the refractive index difference between the internal modes, mode walk-off will occur, resulting in signal distortion and difficulty in demodulation. Studies have shown that at the microscopic level, the angular momentum of electromagnetic waves also has a certain mechanical effect, which will cause the particles on the propagation path to rotate. In addition, the angular momentum of electromagnetic waves can be divided into two parts, one part is called SAM and the other part is called OAM, and in order to facilitate the derivation and analysis, they are represented by *S* and *L*, respectively [26, 27]. For a complete torus, the isophase surfaces are two helical surfaces with an angle of 180 between them, the interferogram of plane wave and spherical wave varies greatly, but the mode orbital angular momentum can still be judged from the spherical wave interferogram.

If the orbital angular momentum is further used in conjunction with polarization, the system capacity can be maximized without increasing the bandwidth. The orbital angular momentum is +2, and the orbital angular momentum of the mode orbital angular momentum crystal is −2.

(1) $$\begin{array}{c} y\left(\alpha ,\beta ,\theta \right)=\left[\begin{array}{ccc} c\alpha -1 & c\beta -1 & c\theta -1\\ c\alpha -2 & c\beta -2 & c\theta -2\\ c\alpha -n & c\beta -n & c\theta -n \end{array}\right]. \end{array}$$

Transmissive helical structures include single-step structures and multistep structures. When conventional plane electromagnetic waves pass through the transmissive helical structure, the thickness of the medium at different positions of the helical structure is different so that the transmitted waves at different positions have a certain degree of thickness. The difference in the wave path difference will lead to different amount of phase change and then form a helical phase factor with exp-i, so this structure can convert ordinary plane waves into vortex waves carrying orbital angular momentum.

(2) $$\begin{array}{c} \left[\begin{array}{cc} c\theta -n & \theta -1\\ \theta +1 & c\theta +n \end{array}\right]\times \left[\begin{array}{cc} 1 & -\theta \\ \theta & 1 \end{array}\right]=\left[\begin{array}{cc} c\theta & -n\\ n & -c\theta \end{array}\right]. \end{array}$$

For HG mode and LG mode, the former has no orbital angular momentum, and on the contrary, the latter has orbital angular momentum and is an eigenstate of orbital angular momentum. The process of their conversion into orbital angular momentum can be seen as the superposition of the two, and it has nothing to do with who is superimposed on whom. Meanwhile, Table 1 is an orthogonal complete pattern basis between them, so one of the two can be arbitrarily selected to expand the other.

Computational holography uses the method of wavefront reconstruction and the computer to simulate the field distribution of electromagnetic waves from the modal number of orbital angular momentum. The key to the whole technology is to load the ordinary electromagnetic wave with orbital angular momentum. Because the orbital angular momentum beam has a helical phase wavefront, the interference fringe pattern generated during interference contains a cross-dislocation structure, and the cross-dislocation structure of the vortex beam is recorded. The phase hologram can be obtained, and then, the fork-shaped grating is engraved by using the medium substrate, which is the holographic plate.

### 3.2. Mechanical Kinematics Analysis

In order to meet the configuration requirements of the manipulator, a connection module is sometimes required to be fixed between two adjacent functional modules. When the configuration of the manipulator needs to be changed, the module needs to be quickly disassembled and assembled. Compared with the beam with uniform polarization, the polarization direction of each point on the cross section of the cylindrical vector beam is different, and the distribution is axisymmetric; in addition, in the light intensity distribution, the OAM light intensity is a structure with a ring center and a dark spot, and the above is the polarization direction of the cylindrical vector beam and the characteristics of the OAM light intensity distribution. Another nonclassical light field is the vortex beam, the wavefront phase of which is distributed in a spiral shape, and the light intensity is also distributed in a ring shape. A typical link model of a reconfigurable manipulator is shown in the text. In order to realize the fixed connection between the two modules and avoid relative sliding, an auxiliary connection module with small mass and reliable fixing effect is used.

(3) $$\begin{array}{c} f\left[t|\theta \left(1\right),\theta \left(2\right),\theta \left(3\right),\ldots ,\theta \left(n\right)\right]=\left[0,-\theta \frac{\left(t\right)}{pi},-\theta \frac{\left(t-1\right)}{pi},-\theta \frac{\left(t-2\right)}{pi},\ldots ,-\theta \frac{\left(t-n\right)}{pi}\right]. \end{array}$$

A vortex electromagnetic wave carrying orbital angular momentum has a helical phase front, if the helical phase front of the vortex electromagnetic wave can be restored to a plane phase front. The information carried by the specific orbital angular momentum state can be extracted from the orbital angular momentum multiplexed light, and the interference generated by other subchannels can be filtered out.

The center wavelength is available in a variety of bands; the tuning range is usually 20 nm; and customized versions with different shapes, bandwidths, and center wavelengths can be provided upon request, and the FBG provided by the user can also be installed in the WTF-200 tunable FBG fiber filter.

In the configuration plane, the swivel joint of Figure 1 serves as the boundary between the configuration planes, has the same function as the connection module, and has no influence on the position of the end point in the configuration plane. Therefore, we take the number of modules in the configuration plane that affect the end position of the robot, that is, the number of rocking modules and moving modules, as the number of degrees of freedom in the configuration plane. A helical fiber Bragg grating (H-FBG) and ytterbium-doped fiber (YDH, Ytterbium, Doped Fiber) FM-FBGs and H-FBG is directly written into the dual-mode fiber (TMF, Two-Mode Fiber).

(4) $$\begin{array}{c} w\left(i-1\right)-w\left(i-t\right)=f\left(\frac{\theta \left(t\right)}{pi},t\right)-f\left(\theta \frac{\left(t-1\right)}{pi},t-1\right)-f\left(\theta \frac{\left(t-n\right)}{pi},t-n\right). \end{array}$$

The ytterbium-doped fiber in the model pumps the signal forward and amplifies it with high reflectivity. FBG1 can be regarded as a wavelength filter, which is used to reflect the oscillating wave of a specific wavelength; here, it is used to reflect the LPol mode with a wavelength. And FBG2 can be regarded as a cavity mirror at the output end, which is used to reflect the redundant wavelengths in the output signal as mixed LP11 modes. The H-FBG in the model can be regarded as the mirror of the input laser source, which can couple the LPol mode and the LP11 mode with wavelength *k* to generate the orbital angular momentum mode.

### 3.3. Neural Network Iteration Hierarchy

Compared with some existing work, for example, at the information sending end, the ordinary electromagnetic wave carrying information is passed through the stepped reflecting surface (assuming that the modal number of the orbital angular momentum generated by the reflecting surface is *l*) so that the azimuth angle increases rotation phase, thereby twisting the ordinary electromagnetic wave propagating in phase on the plane into the OAM vortex wave of the helical phase wavefront. The method proposed in this paper makes the received OAM electromagnetic vortex wave pass through another stepped reflection surface (the modal number of the orbital angular momentum generated by the reflection surface is −l) at the information receiving end so that the azimuth angle is reversed, and the orbital angular momentum vortex wave can be restored to the ordinary electromagnetic wave. For angular connection module, then the kinematic transformation matrix of this module has no variables. Assuming an infinite conductor on the xoy plane, an infinitely long slit of length along the *y*-axis, and a series of plane waves of intensity E0 propagating from the −z region to + *z*, find the electric field strength at point *p* in the xoz plane. First, we use Huygens principle to solve, and then use angle plane spectrum to solve, to compare the conclusions of the two and summarize the basic idea of angle plane spectrum to solve the problem.

(5) $$\begin{array}{c} T_{1-n}^{n-t,1}\left(t,t\left(x\right)\right)=\sqrt{\text{team}\left(t\left(x,x-1\right)\right)}\times \sqrt{\text{team}\left(t\left(x-1,x-1\right)\right)}\times \cdots \times \sqrt{\text{team}\left(t\left(x-t,x-1\right)\right)}. \end{array}$$

It can be seen from the above inference that each parameter in the configuration plane can be obtained, that is to say, the overall value is known, that is, from the starting point of the configuration plane to the end of the configuration plane, the swing module between them is the deflection angle is known, which means that the pose of the center point of the configuration plane becomes known, which limits the movement space of some joints, and the movement range of the entire configuration plane in Figure 2 is limited to a small in the range.

Reference [18] used the mutual orthogonality between OAM vortex waves of different modes and used the number of modes of the orbital angular momentum vortex wave as a modulation parameter. Correspondingly, this paper modulates the information of each channel to the orbital angle of different modes. On the momentum vortex wave, the transmission characteristics of orbital angular momentum are studied, and its modal purity, modal detection, and reception are studied in detail, which is the basis for the follow-up study of vortex wave modal detection and reception. For each identification network, there are the following initialization values: the initial weights of the network are all set to zero; after many simulation experiments, it is found that when the number of hidden layer nodes of the network is initialized to 21, the neural network identification effect can already meet the requirements. When the number of layer nodes is initialized to 31, the identification effect is ideal, so the number of hidden layer nodes is set to 31; the center point of each node of the network takes the value according to the input range of the network, and the input range is [−0.2, 0.2] within the range.

### 3.4. Nonlinear Analysis of Network Data

According to the neural network parameter table and the positive kinematics modeling method of the configuration plane, the relationship transformation matrix of each joint of the manipulator can be obtained, and the mathematical model of the kinematics of the manipulator can be obtained. And it may use MATLAB Robotics Toolbox to model; calculate the position coordinates of the end of the manipulator, given the offsets of each joint; and compare them with the position coordinates calculated by the configuration plane method.

The planar reflection array is composed of units with the same topological structure but different sizes. Using the advantages of the reflection unit in Figure 3, the phase of the electromagnetic wave can be flexibly controlled, and each position can be accurately calculated according to the required model of the orbital angular momentum vortex wave. The incident wave emitted by the feed antenna is irradiated on the plane reflection array, and after the compensation phase provided by the plane reflection array structure is obtained, it is reflected by the phase shift network so that the reflected beam forms a wave with exp(−*jφ*) on the plane reflection array front phase distribution, resulting in an orbital angular momentum vortex beam of mode *l*.

(6) $$\begin{array}{c} T_{1-n}^{n-t,1}\left(t,t\left(x\right)\right)-T_{1-n}^{n-t,1}\left(x,x\left(t\right)\right)=\frac{\text{root}\left(x,t\left(a-1\right)\right)}{1-\text{root}\left(x,t\left(a-1\right)\right)}. \end{array}$$

Due to the narrow working bandwidth of 1-bit reconfigurable artificial metasurfaces, the research on this problem can greatly improve the practical application of 1-bit reconfigurable metasurfaces. The propagating mode causes the power of the transmitting mode to propagate to the adjacent mode: the polarization mode is converted to left-handed circular polarization after passing through the disk. In this paper, a design method of center frequency is proposed. Through experiments, the relative bandwidth of −1 dB gain is 8.4%, which is better than the existing design methods. The existing polarization converters with reconfigurable characteristics can only realize the conversion of specific polarized waves. In this regard, this paper proposes to introduce a varactor diode into a square chamfered unit and realizes the generation of various polarized electromagnetic waves through electrical adjustment without changing the polarization of the incident wave.

## 4. Construction of Data Model Based on Mechanically Reconfigurable Arrays and Neural Networks

### 4.1. Mechanically Reconfigurable Array Configuration Plane Division

Assuming that ports 1 to *N* of the mechanically reconfigurable array are *N* excitation source ports, which are also the response ports of the reconfigurable element, these *N* ports can include any number of polarizations or modes. Assume that ports *N* + 1 to *N* + *M* are the corresponding ports of lumped elements, which can include diodes, inductors, capacitors, and other elements. For these problems, we can abstract active or passive devices into a two-port network. In the simulation, a lumped port is used instead of a full-wave simulation so that a multiport scattering parameter can be obtained. The CNN technology can provide excitation with equal amplitude and phase to each array element, but the orbital angular momentum vortex beam of different modes of broadband and circular polarization is not uniform. Compared with CNN technology, this paper can generate orbital angular momentum vortex waves of different modes by adjusting the rotation angle of the array element around its own axis so as to realize the mechanical reconfigurability of the device.

(7) $$\begin{array}{c} \left\{\begin{array}{c} h\;\sin\left(i,j\right)=\left(h-1\right)\sin\left(i+1.j+1\right),\\ h\;\cos\left(i,j\right)=\left(h-1\right)\cos\left(i+1.j+1\right). \end{array}\right. \end{array}$$

It receives the information from the input layer and processes it and maps the input data to the hidden layer space. The mapping in this process is a nonlinear transformation. The function that performs nonlinear transformation in the hidden layer is called the activation function of the network. Generally, it is a nonlinear and positive decay function (called radial basis function) that is symmetrical to the radial center, so the network has the characteristics of local function approximation, and if the distance between the input data and the function center point is smaller, the network will be more sensitive to this input variable, and the better the function approximation effect.

There is a relative delay between adjacent parts of the beam, thereby achieving the effect of wavefront distortion. The output layer of the network receives the data processed by the hidden layer, linearly adds the output data of the hidden layer, and output the final result from the network. The threshold constant vector is zero in the network in Figure 4.

At present, in the generation method of OAM, the realization of CNN array antenna is relatively difficult, and the verification conditions are not yet available. However, the CNN microstrip antenna generally has the characteristics of high *Q* value of common resonant antennas, which makes the change of frequency have a decisive impact on its input impedance, so its working frequency band is narrow, which becomes the microstrip antenna of CNN. In order to verify the principle, an 8-element circular array operating at 3.4–4.7 GHz is simulated and processed. The array is excited by a one-to-eight equal-amplitude in-phase microstrip line feed network, and the output ports are, respectively, the same as eight identical single arms. The helical antenna units are connected, and the orbital angular momentum vortex beams of different modes are generated by adjusting the rotation angle of each single-arm helical antenna unit.

### 4.2. Multimodal Algorithm Equation Solution

Wireless energy transfer based on reconfigurable metasurfaces is a new means of flexibly transferring wireless energy according to external dynamic demands. The OAM vortex electromagnetic wave array antenna designed in this paper is used for the transmitting end of the mobile communication system. Compared with the conventional coupled wireless energy transmission, it has a longer transmission distance and greater flexibility. From the analysis of achievability and transmission efficiency, 2-bit is the first choice for digitizing electromagnetic focusing surfaces. In this paper, a U-shaped two-arm asymmetric slotted unit is proposed, using two PIN diodes to achieve 90°, 180°, and 270° phase differences. Based on this unit, a 12 × 12 two-bit electromagnetic focusing surface is realized. The near-field energy focusing effect is obtained in the experiment, and the flexible transfer of energy is verified by the antenna transmission simulation.

(8) $$\begin{array}{c} \langle \begin{array}{cc} c\times \;\sin\left(i,j\right) & \alpha \left(i-1\right)\\ i-1 & -c\times \;\sin\left(i,j\right) \end{array}\rangle ⟶\langle \begin{array}{cc} c\times \;\exp\left(i,j\right) & i-1\\ i & -c\times \;\exp\left(i,j\right) \end{array}\rangle . \end{array}$$

In the complex configuration of the robot, for the design *H* joint configuration, positive kinematics is one of the typical problems to be solved. There are many existing methods for finding positive kinematics. In order to find the position and posture of adjacent joints in the configuration of the manipulator, the D-H algorithm provides a systematic and convenient method for the robot designer. In the D-H algorithm, the coordinate system is first established for each robot module, and the adjacent coordinate systems are connected so that the relationship transformation matrix of the adjacent joints in Table 2 can be easily expressed, and then, the position and attitude of each module can be expressed. The vortex beam virtual concrete means that the OAM beam has a helical phase characteristic in a plane perpendicular to the propagation direction. The OAM has infinitely many modes, and each mode is orthogonal to each other, which provides natural conditions for the communication and detection of vortex waves. In theory, vortex waves can increase communication capacity infinitely. The method of generating and transmitting in the fiber simplifies the optical structure and has higher phase purity. The vortex beam is obtained by superposition of the corresponding order vector modes in the corresponding fiber, and its phase purity is higher. We know that vortex beams can carry independent data streams in different orthogonal modes.

When the signal is input from the input terminal and enters the *H*. After FBG, LPs mode, and LP, the l-modes are cross-coupled at wavelength *h*, where a portion of the energy is reflected and the remaining energy continues to be transmitted forward. After the residual signal energy enters the YDF, it is amplified and continues to transmit forward under the combined action of the Pump signal and the YDF. At FBG1, LPol in the signal is 100% completely reflected at wavelength *h*, while LP11 passes. The reflected LPol mode is transmitted to the left, when entering *H*. During FBG, cross-coupling with the remaining LP11 modes occurs and propagates to the right. This part of the energy is also amplified when passing through YDF and continues to be transmitted to the right, after passing through FM-FBGl and FM. After FBG2, output from the output terminal, this part of the signal is a vortex beam carrying orbital angular momentum.

### 4.3. Orbital Angular Momentum Data Normalization

In order to realize the directional radiation characteristics of the orbital angular momentum of the planar single-armed helix antenna, a dielectric substrate 3 with the same material as the dielectric substrate 1 is placed at a distance of 35 mm (about a quarter of the central working wavelength) below the planar single-armed helix. The radius is 150 mm, the thickness is 1 mm, and the upper surface of the dielectric substrate 3 is set as PEC, which is used as the reflection floor of the planar single-arm helical antenna to suppress the bidirectional radiation of the antenna. Because the OAM vortex wave with mode number 0 is actually an ordinary electromagnetic wave and does not have the characteristics of helical phase wavefront, the simulation results also found that the transmission coefficient between the 0 modes is larger than that between the 0 modes. It is worth noting that when applying the OAM transceiver link to an actual communication system, if the system includes a mode 0 transceiver antenna, an attenuator should be used before to keep its transmission amplitude and orbital angular momentum vortex wave within the same range within the same level. The radius of the inner core is 0.65 mm and the height is 36 mm, the upper end is connected to the upper surface of the dielectric substrate 2, and the lower end is connected to the upper surface of the dielectric substrate 3.

(9) $$\begin{array}{c} \frac{R_{\text{redirst}}^{i+j}\left(f\left(i,j\right)\right)}{\left[\begin{array}{cc} 1-\sqrt{f\left(t\right)} & 1\\ 1 & -1-\sqrt{f\left(t\right)} \end{array}\right]}=\frac{R_{\text{redirst}}^{i+j}\left(a,b\right)}{\left[\begin{array}{cc} 1-a & 1\\ 1 & -1-b \end{array}\right]}. \end{array}$$

At the initial moment, the robot is in a static state, and at this time, the transformation relationship matrix of each module joint of the robot can be initialized, that is, it is described by the specific values of the four parameters. During the movement of the robot, if any one parameter changes or is different, the transformation relation matrix 7 will change, model the metasurface element in HFSS, add a lumped port at the position where the diode equivalent circuit needs to be added, and set its impedance as Zref.

The flat single-arm spiral is printed on the upper surface of the dielectric substrate 1 with a radius of 33 mm and a thickness of 1 mm. The dielectric substrate in Figure 5 adopts F4B, its relative permittivity is 2.65, and the loss tangent is 0.003. The tail of the flat single-arm helix is made sharp, and a chip resistor with a resistance value of 160 is placed at the end to reduce the tail current reflection on the helical arm and reduce the “truncation” effect. A dielectric substrate 2 with a radius of 10 mm and a thickness of 2 mm is placed next to the lower surface of the dielectric substrate 1.

The material in Table 3 of the dielectric substrate 2 is the same as that of the dielectric substrate 1, and the lower surface of the dielectric substrate 2 is set as a PEC. The purpose is to achieve impedance matching, thereby further broadening the working frequency band of the antenna.

## 5. Application and Analysis of Multimodal Orbital Angular Momentum Data Model Based on Mechanically Reconfigurable Array and Neural Network

### 5.1. Inverse Solutions of Mechanically Reconfigurable Array Functions

In this paper, the multiple vortex electromagnetic wave generators are realized by two methods: continuous and discrete. First, in order to simulate the characteristic that the phase shift of conventional metasurface elements can be continuously adjusted, a reconfigurable element loaded with varactors is proposed to realize the orbital angular momentum vortex wave generator. A 16 × 16 reconfigurable metasurface operating at 5.0 GHz was designed, and four vortex electromagnetic waves with different transmission directions and different modes were measured experimentally.

(10) $$\begin{array}{c} \underset{\text{i,j}<1}{\sum }R_{\text{redirst}}^{i+j}\left(\alpha \left(i,j\right)\right)+R_{\text{redirst}}^{i+j}\left(\alpha \left(i-1\right)\alpha \left(j-1\right)\right)+\cdots +R_{\text{redirst}}^{i+j}\left(\alpha \left(1,1\right)\right)=\frac{\sin\left(\alpha \left(i,j\right)\right)}{\cos\left(\alpha \left(i,j\right)\right)}. \end{array}$$

Furthermore, in order to simplify the design of the electrically tunable vortex wave generator, this paper proposes to use a 1-bit reconfigurable metasurface to generate vortex waves. The calculation process of the compensation phase calculation method for 1-bit vortex wave generation is given. A 12 × 12 1-bit digital surface was designed, and vortex electromagnetic waves in different modes were measured experimentally.

(11) $$\begin{array}{c} \left[\begin{array}{c} R_{\text{redirst}}^{i+j}\left(\theta \left(i,j\right)\right)\\ R_{\text{redirst}}^{i+j}\left(\beta \left(i,j\right)\right)\\ R_{\text{redirst}}^{i+j}\left(\alpha \left(i,j\right)\right) \end{array}\right]=\left[\begin{array}{c} \sin\;\theta \left(i,j\right)\\ \sin\;\beta \left(i,j\right)\\ \sin\;\alpha \left(i,j\right) \end{array}\right]. \end{array}$$

The six-degree-of-freedom manipulator includes seven modules from the base coordinate to the end: the rotation module, the swing module, the connection module, the swing module, the rotation module, the wrist swing module, and the end rotation module. According to the definition and method of the configuration plane, after calculation, one configuration plane cannot meet the attitude requirements of the manipulator. According to the method of two configuration planes to match and calculate, the two configuration planes can meet the configuration attitude requirements.

In addition to the method of generating orbital angular momentum electromagnetic waves in the form of antenna shaping such as helical paraboloids, the array antenna in Figure 6 is also another method that can generate orbital angular momentum waves. Generally, it can be adjusted by adjusting the feed between each adjacent array element so as to realize the emission of vortex electromagnetic waves carrying different modal values, and this structure can meet the requirements of generating multimodal orbital angular momentum. Arranging several antenna elements and other rules, with the help of electromagnetic wave interference and superposition theory, controls the feed phase difference between each array element so that the energy radiated by the electromagnetic field can be redistributed in space, and the uneven distribution of space energy can be realized. That is, the field increases in some areas and decreases in some areas.

### 5.2. Simulation of Multimodal Orbital Angular Momentum Data Model

A capacitive reactance can be generated between the part of the *L*-shaped probe of the orbital angular momentum antenna that is parallel to the metal patch and the metal patch, and an inductive reactance can be generated between the part of the probe perpendicular to the metal patch and the metal patch. The inductive reactance interaction can make the internal field of the air medium resonate, which can make the antenna have the characteristics of multiband or wideband. When the *L*-shaped probe is connected to the coaxial feeder, a corresponding alternating electric field will be generated on the probe. At the same time, the electric field will generate a changing magnetic field, and the field strength directions of the two fields are perpendicular to each other. When the magnetic field lines pass through the microstrip patch, the magnetic field will generate a changing electric field. Finally, reflected off the metal ground plate, the changing electromagnetic field is radiated to the outside space in this way.

(12) $$\begin{array}{c} \frac{\left[\begin{array}{ccc} a+bi & a & 1\\ a & a+bj & a\\ 1 & a & a+bk \end{array}\right]}{w\left(a\right)+w\left(b\right)+w\left(c\right)}=\left[\begin{array}{ccc} a & a\;\cos\;i & 1\\ -a\;\cos\;i & b & -a\;\cos\;i\\ 1 & a\;\cos\;i & c \end{array}\right]. \end{array}$$

However, there are some problems in the measurement results compared with the simulation results. It can be seen that the helix on the measurement observation surface is not smooth and flat. The main reason for this problem is that the sampling interval is too large. The effect of the measured distance and the phase distribution of the electric field will be closer to the simulation results. However, the measurement results are in good agreement with the simulation analysis. The mapping between the hidden layer and the output layer is linear, that is, the linear sum of the hidden layer output and the output weight. Using the network to approximate a function or identify a model greatly increases the learning speed and effectively avoids local minima. A large number of experiments have proved that the network meets the needs of real-time control. Since the phase plate has a helical surface structure, when the wave beam passes through the phase plate, the difference in the path difference of the beam will cause different phase changes so that the transmitted beam changes from a normal electromagnetic wave to a vortex electromagnetic wave with a helical phase structure. Vortex beams with various modal values of orbital angular momentum can be generated by changing the step height of the spiral phase plate steps.

It can be seen that the electric field phase distribution on the observation surface presents a counterclockwise helical structure. The mode *l* = 1 in Figure 7 is a one-armed helix, and the mode *l* = 2 and mode *l* = 3 are two-arm and three-arm, respectively; the electric field amplitude distribution also presents a counterclockwise helical shape, when the modes *l* = 1, *l* = 2, and mode *l* = 3 are a double-armed, four-armed, and six-armed helical structure, respectively.

(13) $$\begin{array}{c} \tanh\left(w\left(a\right)+w\left(b\right)+w\left(c\right)\right)=\left\{\begin{array}{c} \sum \frac{w\left(i\right)}{w\left(i\right)-1},i>1,\\ \frac{w\left(a\right)+w\left(b\right)+w\left(c\right)}{\sum w\left(i\right),i<1}. \end{array}\right. \end{array}$$

Based on the theoretical basis of the rectangular patch antenna, an improved method of broadband antenna is proposed. The array antenna proposed in this paper shows good performance in its corresponding operating frequency band and can generate vortex electromagnetic waves carrying multiple modes of orbital angular momentum, of which the maximum generated mode values are 1, 2, and 3, and it focuses on the array feeding methods such as phase control technology and high-speed RF switching technology, as well as the integration of circular polarization theory into the design of vortex electromagnetic wave array antenna. Further observing the characteristics of the 3D pattern, we can see that the 3D patterns in different modes have a central concave structure, and with the increase of the orbital angular momentum mode, the concave in the middle of the far-field radiation pattern becomes more and more is large, which is consistent with the theoretical radiation characteristics of orbital angular momentum vortex waves in each mode. It can be seen from the results that the rotation curves of the electric field phase distribution diagrams along the *x* and *y* directions of the same modal orbital angular momentum vortex beam have a phase difference of 90. It can be seen that the orbital angular momentum vortex beam generated by the 8-element array is circularly polarized. Compared with references [16, 17], the above measurement process shows that the modal number of OAM vortex waves can be easily and effectively detected by using the phase gradient method. In addition, the more the number of receiving probes, the smaller the error of the result and the higher the accuracy of the test result.

### 5.3. Example Application and Analysis

The example part uses ANSYS HFSS to design several multimode orbital angular momentum vortex electromagnetic wave microstrip array antennas operating in the x-band, L-band nozzle, and 245 GHz frequency band and gives the different orbital angular momentum modal value vortices generated by the array antenna. The simulation experiment utilizes the far-field phase characteristics of the antenna itself to realize the mechanical reconfigurable characteristics of the device and at the same time simplify the feed network and validity and correctness of the idea. On this basis, the modal purity, detection method, and reception of orbital angular momentum are studied accordingly. It is proved that the array antenna can generate vortex electromagnetic waves with different modal values of orbital angular momentum under the conditions of simulation experiments, dividing the manipulator into three configuration planes, where the base coordinates are contained in the first configuration plane and the end of the manipulator is contained in the third configuration plane. Since the end of the manipulator is included in the third configuration plane, and the target point of the manipulator has been given, we set the *X*-axis direction of the third configuration plane as the normal direction of the configuration plane, and then, the first poses of the three configuration planes are also determined.

(14) gh,k,l−sinhxi−xj+coshxi−xjNoi−oj=0.

The length of the microstrip line from port 1 to port 3 is longer than the length of the microstrip line from port 1 to port 2, so there is a 45-leaf bit delay from port 3 compared to port 2; the feeding principle of port 4 and port 5 is to use in the same way, 90 can be implemented on port 4 phase delay, while port 5 has a 135-bit delay. The lower half of the feed network is obtained by rotational symmetry with the center of the upper half. The phase shift reduces the total area of the feed network accordingly. The structure of the microstrip feed network and the design parameters of the array antenna are as described in the text.

At the basic operating frequency, each element of the time-transformed array is excited with a unit amplitude and the same phase, but each array element in Figure 8 is excited separately in sequence, that is, each array element only has to turn on for a period of time shovel, IV, where tile is the total time to turn on IV arrays sequentially. Coaxial feed microstrip line function is ram, feed port −4 ram, and uses 50 n SMA connectors in order to maintain good impedance matching of the feed network. A microstrip array antenna   mm with a single feed channel angular momentum of 4% is fabricated on a dielectric substrate with a thickness of 6. The radius of the dielectric substrate is R-255 ram. The material is FR4. Its relative permittivity *e* is 44.

The electric field strength near the direction of the propagation axis of the beam is very weak, and even the phenomenon of hollow zero occurs. This phenomenon is caused by the different phases of each pair of adjacent array elements. It can also meet the requirements of wireless communication signal transmission by arranging multiple nonpolarized antennas in a relatively large space. The hollow area in Figure 9 is too small depending on the array antenna radius and the orbital angular momentum mode. The hollow area is too small so that an accurate estimation of the orbital angular momentum cannot be obtained, and in order to realize orbital angular momentum multiplexing communication, it is necessary to achieve breakthroughs in the corresponding key technologies: generation of high-quality vortex beams carrying OAM, channel coding and modulation, free space transmission characteristics, and receiving end beam separation and detection, etc. The single-feed orbit angular momentum microstrip array antenna electric field magnitude diagram can be seen and obtained using the feed network. After the phase delay of the array element, the rotating phase wavefront of the orbital angular momentum mode *L* ± *l* is clearly displayed, and the beam appears hollow along the propagation direction of the electromagnetic wave, which indicates that the orbital angular momentum mode island *l* helical phase distribution has been successfully generated by the orbital angular momentum array antenna.

## 6. Conclusion

Based on the theory of mechanically reconfigurable array and neural network, this paper introduces and compares the generation methods of orbital angular momentum vortex waves in detail and makes a method for generating orbital angular momentum vortex waves from circular array antennas in the microwave radio frequency section. Using the far-field phase characteristics of the single-armed helical antenna, that is, when the single-armed helical antenna rotates around its own axis, the amplitude of the electric field at the far-field remains unchanged, and the phase change is consistent with the rotation angle. Comparing the results of different digital quantizations, it is determined that 2-bit is the best choice for both achievability and efficiency. The advantage of this method is that the antenna configuration required by the spatial multiplexing technique is relatively low, and there is no high spatial correlation between the transmitter and receiver antenna wells. The broadband circularly polarized single-arm helical antenna with the working frequency band of 1.73–9 GHz is simulated and designed, and eight identical single-armed helical antennas are used to form a circular ring array antenna; the feeding network is simplified from a general power divider phase shifter to a power divider, which provides 8 array elements with excitation of equal phase and the same amplitude. The mathematical function describing a Gaussian beam is a paraxial approximation of the Helmholtz equation (a type of small-angle approximation). This solution has the form of a Gaussian function that represents the complex amplitude of the electric field component in the beam. Finally, the reflection coefficient, axial ratio, and far-field pattern of the array in each mode are tested experimentally, which are consistent with the simulation results; the electric field amplitude and helical phase distribution of the array are tested under near-field and far-field conditions, and far-field patterns are consistent with the results of theoretical analysis, which proves the correctness and effectiveness of the method. Correspondingly, the far-field pattern of the high-frequency band of the traditional method is not very ideal, and further research is needed to minimize the influence of the outer ring antenna on the inner ring antenna. Therefore, with the progress made in machine vision, the computational method in this paper may need to be further improved and perfected.

## Figures and Tables

**Figure 1:** 3D analysis of mechanical kinematics rotary joint.

**Figure 2:** Neural network iterative hierarchy topology.

**Figure 3:** Plane distribution of network data nonlinear configuration.

**Figure 4:** Two-dimensional distribution of mechanically reconfigurable array configuration plane division.

**Figure 5:** Normalized orbital angular momentum data of planar single-arm helix.

**Figure 6:** Inverse solution distribution of mechanically reconfigurable array function.

**Figure 7:** Multimodal orbital angular momentum logic loop.

**Figure 8:** Parameter distribution of orbital angular momentum electric field amplitude characteristic.

**Figure 9:** Orbital angular momentum modal value vortex electromagnetic wave gain distribution.

**Table 1:** Reconfigurable array description.

Multiplexed index	The configuration plane	Mechanical kinematics	Rotary joint case	3D analysis range
**1**	11.77	Connection module	0.87	[−1, 1]
**2**	32.08	Rocking module	0.40	[−1.21, 0.981]
**3**	48.34	Rocking module	0.45	[−1, 1.224]
**4**	39.40	Combination module	0.77	[−0.341, 1.1]
**5**	46.61	Connection module	0.43	[−0.31, 1.21]
**6**	44.54	Connection module	0.11	[−1.21, 1.51]
**7**	28.23	Combination module	0.12	[−0.571, 0.981]
**8**	10.82	Combination module	0.038	[−0.812, 1.114]

**Table 2:** Multimodal orbital angular momentum algorithm steps.

Algorithm step number	Multimodal orbital angular content
In the complex configuration *w*(*i*)	Static int interspacef = brick_width;
For the robot designer *a*^2^+*b*^2^	Node_pos = [(1, 0), (0, 1), (2, 1), (1, 2)]
The d-h algorithm provides *p*(*x*, *x*(*t*))	Bbox_args = dict(boxstyle = “round”)
A Θ(*t*, *t* − 1, *t*+1) convenient method *w*(*i*) − 1	Head and tail patch, respectively.
In the configuration of the min.(*s*)	Xycoords: str, artist, transform
Posture of adjacent joint *w*(*a*)+*w*(*b*)+*w*(*c*)	Import matplotlib.pyplot as plt
In order to find the position max(*i*, *j*)	Import numpy as np
For finding *w*(*j* − 1) positive kinematics	From matplotlib.lines import line2d
*h*(*x*(*i*) − *x*(*j*)) to be solved	Arrowprops = dict(patcha = an1)
$1-\sqrt{g\left(t\right)}$ of the robot for the design h	Patchb = an2, matplotlib.patch.
*o*(*i*) − *o*(*j*) is one of the typical problems	Connectionstyle = “arc3,rad = 0.2″
Joint configuration and *q*(*t*, *t*(*x*)) kinematics	#color = “red”, patch instance

**Table 3:** Orbital angular momentum parameters table.

Momentum parameter symbol	Physical meaning analysis
*I*	Vortex beam real part
*J*	Vortex beam imaginary part
*X*	Coordinate direction
*Y*	Coordinate direction
*Z*	Coordinate direction
FBG	Fiber Bragg grating
FM	Frequency modulation
TRL	Thru reflect line
HFSS	High-frequency structure simulator
PEC	Perfect electrical conductor

## Data Availability

The data used to support the findings of this study are available from the corresponding author upon request.
